# Baseline CD4 Cell Counts of Newly Diagnosed HIV Cases in China: 2006–2012

**DOI:** 10.1371/journal.pone.0096098

**Published:** 2014-06-05

**Authors:** Houlin Tang, Yurong Mao, Cynthia X. Shi, Jing Han, Liyan Wang, Juan Xu, Qianqian Qin, Roger Detels, Zunyou Wu

**Affiliations:** 1 Division of Integration and Evaluation, National Center for AIDS/STD Control and Prevention, Chinese Center for Disease Control and Prevention, Beijing, China; 2 Department of Epidemiology, School of Public Health, Harvard University, Boston, Massachusetts, United States of America; 3 Division of Epidemiology, National Center for AIDS/STD Control and Prevention, Chinese Center for Disease Control and Prevention, Beijing, China; 4 Department of Epidemiology, School of Public Health, University of California at Los Angeles, California, United States of America; Istituto Superiore di Sanità, Italy

## Abstract

**Background:**

Late diagnosis of HIV infection is common. We aim to assess the proportion of newly diagnosed HIV cases receiving timely baseline CD4 count testing and the associated factors in China.

**Methods:**

Data were extracted from the Chinese HIV/AIDS Comprehensive Response Information Management System. Adult patients over 15 years old who had been newly diagnosed with HIV infection in China between 2006 and 2012 were identified. The study cohort comprised individuals who had a measured baseline CD4 count.

**Results:**

Among 388,496 newly identified HIV cases, the median baseline CD4 count was 294 cells/µl (IQR: 130–454), and over half (N = 130,442, 58.8%) were less than 350 cells/µl. The median baseline CD4 count increased from 221 (IQR: 63–410) in 2006 to 314 (IQR: 159–460) in 2012. A slight majority of patients (N = 221,980, 57.1%) received baseline CD4 count testing within 6 months of diagnosis. The proportion of individuals who received timely baseline CD4 count testing increased significantly from 20.0% in 2006 to 76.9% in 2012. Factors associated with failing to receiving timely CD4 count testing were: being male (OR: 1.17, 95% CI: 1.15–1.19), age 55 years or older (OR:1.03, 95% CI: 1.00–1.06), educational attainment of primary school education or below (OR: 1.30, 95% CI: 1.28–1.32), infection with HIV through injection drug use (OR: 2.07, 95% CI: 2.02–2.12) or sexual contact and injection drug use (OR: 1.87, 95% CI: 1.76–1.99), diagnosis in a hospital (OR: 1.91, 95% CI: 1.88–1.95) or in a detention center (OR: 1.75, 95% CI: 1.70–1.80), and employment as a migrant worker (OR:1.55, 95% CI:1.53–1.58).

**Conclusion:**

The proportion of newly identified HIV patients receiving timely baseline CD4 testing has increased significantly in China from 2006–2012. Continued effort is needed for further promotion of early HIV diagnosis and timely baseline CD4 cell count testing.

## Introduction

CD4 cell count is a major indicator of human immunodeficiency virus (HIV) infection disease progression [1], [2]. Patients who receive a late diagnosis, defined as a baseline CD4 cell count<200 cells/µl, have significantly poorer responses to antiretroviral therapy (ART) and worse prognoses [3], [4], [5], [6]. The proportion of patients who present late to diagnosis and treatment remains unacceptably high [7], [8], [9], [10]. Internationally, the observed proportion of patients with late diagnoses is stable or worsening [7]. Although it is recommended that CD4 cell count testing should be carried out promptly after diagnosis, many patients fail to receive on-time testing [11], [12]. In the United States, an ongoing outpatient study in eight cities found that 78% of patients had a measured CD4 count within 3 months of HIV diagnosis [7]. This proportion was significantly lower in developing countries. Studies in Thailand, Vietnam, and South Africa reported that only 34%, 49%, and 62.6% of patients, respectively, received CD4 count assessment with 6 months of HIV diagnosis [13], [14], [15].

In 2002, China implemented the National Free Antiretroviral Therapy Program (NFATP) to address the issue of poor access to HIV/AIDS treatment. Patients who meet the national treatment criteria of a CD4 count ≤200 cells/µl (revised to ≤350cells/µl in 2008) are eligible for ART at no cost to the patient [16]. The program has contributed to a dramatic reduction in mortality among patients receiving HIV treatment [17]. In order to expand NFATP coverage, the government has increased HIV screening access, leading to a rise in the number of people diagnosed with HIV [18]. After the diagnosis of HIV infection, timely CD4 cell count testing is a crucial step in determining whether the patient meets criteria for ART initiation and engaging the patient in appropriate care and treatment [19], [20]. From 2007, the national HIV/AIDS program set quantitative targets of core indicators to monitor progress in key areas of HIV work. From 2007 to 2009, the proportion of CD4 cell count monitoring for people diagnosed with HIV and AIDS increased from 45.3% and 10.1% in 2007 to 54.2% and 62.5% in 2009, respectively [21].

However, past studies have indicated that many patients are lost or delayed along the continuum of care. A study in Guangxi and Yunnan found that only 37% of patients who were diagnosed with HIV from 2005 to 2009 received baseline CD4 testing within 6 months [20]. The proportion increased dramatically from 7% in 2005 to 62% in 2009. A separate study noted that in 2009, approximately 30% of the ART-initiated patients who received baseline CD4 testing had CD4 <50 cells/µl, indicating that many patients were being diagnosed and treated late [22], [23]. Prompt baseline CD4 testing is a critical step in successful linkage to HIV treatment.

By using data extracted from the Chinese HIV/AIDS Comprehensive Response Information Management System (CRIMS) [24], we aimed to identify trends in the proportion of individuals who received timely baseline CD4 cell count testing within 6 months of HIV diagnosis in China from 2006 to 2012. We also sought to determine changes in median baseline CD4 cell counts over time and factors associated with failing to receive CD4 cell count testing.

## Methods

### Data source

Data were collected from CRIMS, a web-based real-time database system managed by the National Centre for AIDS/STD Control and Prevention (NCAIDS), Chinese Center for Disease Control and Prevention (CDC). CRIMS was developed in 2005 and has previously been described elsewhere [24]. Local CDC staffs, who are trained on data upload and management, create electronic records in CRIMS for each patient who tests positive for HIV. Staffs receive annual refresher training. Patient records contain information on demographic characteristics, contact information (including both permanent and temporary residential addresses), sexual and drug use risk behaviors, likely transmission routes, medical histories, and laboratory test results [24]. For this study, we included all adult individuals (over 15 years old) who received a confirmed HIV diagnosis between January 1, 2006 and December 31, 2012. All HIV screening is done in accordance with national HIV policy. Provider-initiated testing and counseling (PITC) has been in place in hospitals since 2007.

### Data analysis

The primary outcome of interest was the proportion of newly diagnosed HIV/AIDS individuals who received baseline CD4 cell count testing within 6 months of diagnosis. Data were described by the median (interquartile range, IQR) and the distribution across four CD4 cell count categories (<200, 200–349, 350–500, and ≥500). Demographic characteristics were analyzed using chi-squared statistics for dichotomous and categorical variables. Univariate and multivariate logistic regression models were used to assess the factors associated with not receiving a timely CD4 cell count. Variables with p<0.10 under univariate analysis were retained for multivariate modeling using stepwise selection, and 95% confidences intervals were estimated using these models. Results with a two-sided p<0.01 were considered statistically significant. All data analyses were performed using SAS Version 9.3 (SAS Institute, Cary, NC, USA).

### Ethics statement

This study was a secondary data analysis using existing Chinese government HIV/AIDS CRIMS data. All subjects signed a general informed consent upon enrollment to CRIMS indicating that their data, after removing personal identifiers, could be used in statistical analyses and/or epidemiological research studies. Therefore, no additional study specific informed consent was necessary for this current study. Patient records and information were de-identified prior to analysis. This study protocol was reviewed and approved by the Institutional Review Board of the National Center for AIDS/STD Control and Prevention, Chinese Center for Disease Control and Prevention (approval #X130205248).

## Results

Between January 1, 2006 and December 31, 2012, there were 394,294 individuals newly diagnosed with HIV infection in China. Patients under 15 years of age (N = 5,798) were excluded from the study cohort. Of the remaining 388,496 newly diagnosed individuals, 221,980 (57.1%) patients received a baseline CD4 cell count within 6 months of HIV diagnosis over the six-year study period (Table 1).

**Table 1:** Baseline CD4 cell counts (within 6 months of diagnosis) of HIV individuals in China: 2006–2012.

	2006	2007	2008	2009	2010	2011	2012	Total
Total No.	35087	40491	47675	54552	58109	71166	81416	388496
No. (%) of subjects with baseline CD4 cells counts within one year								
<15 days	3812 (10.9)	7021 (17.3)	12038 (25.3)	16332 (29.9)	20544 (35.4)	29437 (41.1)	37561 (46.1)	126745 (32.6)
<30 days	4608 (13.1)	8472 (20.9)	14538 (30.5)	20172 (37.0)	25372 (43.7)	36712 (51.6)	46753 (57.4)	156627 (40.3)
<90 days	5893 (16.8)	10949 (27.0)	18340 (38.5)	25434 (46.6)	32467 (55.9)	46623 (65.5)	57773 (71.0)	197479 (50.8)
<180 days	7030 (20.0)	13125 (32.4)	21122 (44.3)	29078 (53.3)	37081 (63.8)	51957 (73.0)	62587 (76.9)	221980 (57.1)
Median (IQR) baseline CD4 cell count	221(63–410)	252(80–429)	280(106–448)	287(116–454)	295(130–459)	299(140–454)	314(159–460)	294(130–454)
No. (%) of subjects with CD4 cell counts (cells/µl)								
<200	3298 (46.9)	5552 (42.3)	7851 (37.2)	10620 (36.5)	12751 (34.4)	17266 (33.2)	19244 (30.7)	76582 (34.5)
200–349	1476 (21.0)	2941 (22.4)	5062 (24.0)	6858 (23.6)	9062 (24.4)	12877 (24.8)	15584 (24.9)	53860 (24.3)
350–499	1066 (15.2)	2299 (17.5)	4092 (19.4)	5802 (20.0)	7800 (21.0)	11691 (22.5)	15241 (24.4)	47991 (21.6)
≥500	1190 (16.9)	2333 (17.8)	4117 (19.5)	5798 (19.9)	7468 (20.1)	10123 (19.5)	12518 (20.0)	43547 (19.6)

The number of newly identified HIV cases with measured baseline CD4 counts more than doubled between 2006 and 2012, increasing from 35,087 to 81,416. The proportion of newly diagnosed individuals who received a baseline CD4 cell count test within 6 months increased from 20.0% in 2006 to 76.9% in 2012. National policies recommend CD4 cell count testing within 14 days after diagnosis of HIV infection. Our study found that the proportion of newly diagnosed individuals who received baseline CD4 cell count testing within 14 days increased from 10.9% in 2006 to 46.1% in 2012 (Table 1).

The median baseline CD4 cell count of individuals who received timely testing over the study period was 294 cells/µl (IQR: 130–454). Over half of the patients (N = 130,442, 58.8%) had baseline CD4 cell counts <350 cells/µl, and 76,582 patients (34.5%) had baseline CD4 cell counts <200 cells/µl. Less than a quarter of patients (N = 43,547, 19.6%) had baseline CD4 cell counts ≥500 cells/µl (Table 1).

The median baseline CD4 cell count increased slightly by each calendar year over the study period from 221 cells/µl (IQR: 63–410) in 2006 to 314 cells/µl (IQR: 159–460) in 2012. The percentage of individuals with baseline CD4 cell counts <200 cells/µl, indicating advanced disease, decreased from 46.9% in 2006 to 30.7% in 2012. The percentage of individuals diagnosed with baseline CD4 cell counts ≥500 cells/µl, indicating a recent acquisition of HIV infection, has remained relatively stable (Table 1).

Characteristics associated with receiving baseline CD4 cell count testing within 6 months were being female, being married, having attained middle school education or higher, having acquired HIV through male-to-male sexual contact or commercial blood plasma donation, and being diagnosed with HIV infection at a voluntary counseling and testing (VCT) clinic (Table 2). A total of 34,248 newly diagnosed individuals (8.8%) died within 6 months after HIV diagnosis. Of these individuals, 23,661 (69.1%) had not received CD4 cell count testing.

**Table 2:** Factors associated with baseline CD4 cell counts (within 6 months of diagnosis) of HIV individuals in China: 2006–2012, based on multivariate logistic regression analysis.

	No. of new cases	No. (%) of subjects with baseline CD4 cell count	Unadjusted OR (95% CI)	P-value	Adjusted OR (95% CI)	P-value
Year of HIV diagnosis						
2006	35087	7030 (20.0)	1.00		1.00	
2007	40491	13125 (32.4)	0.52 (0.51–0.54)	<0.01	0.57 (0.55–0.59)	<0.01
2008	47675	21122 (44.3)	0.32 (0.31–0.33)	<0.01	0.39 (0.38–0.40)	<0.01
2009	54552	29078 (53.3)	0.22 (0.21–0.23)	<0.01	0.28 (0.27–0.29)	<0.01
2010	58109	37081 (63.8)	0.14 (0.14–0.15)	<0.01	0.19 (0.18–0.20)	<0.01
2011	71166	51957 (73.0)	0.09 (0.09–0.10)	<0.01	0.13 (0.12–0.13)	<0.01
2012	81416	62587 (76.9)	0.08 (0.07–0.08)	<0.01	0.11 (0.10–0.11)	<0.01
Gender						
Female	113340	67460 (59.5)	1.00		1.00	
Male	275156	154520 (56.2)	1.15 (1.13–1.16)	<0.01	1.17 (1.15–1.19)	<0.01
Age (years)						
15–24	58323	31195 (53.5)	1.00		1.00	
25–34	132737	70982 (53.5)	1.00 (0.98–1.02)	0.96	0.82 (0.80–0.84)	<0.01
35–44	101295	58885 (58.1)	0.83 (0.81–0.85)	<0.01	0.80 (0.78–0.82)	<0.01
45–54	43726	28773 (65.8)	0.60 (0.58–0.61)	<0.01	0.80 (0.78–0.83)	<0.01
55+	52415	32145 (61.3)	0.73 (0.71–0.74)	<0.01	1.03 (1.00–1.06)	0.03
Marital status						
Single, divorced, or widowed	175776	101301 (57.6)	1.00		1.00	
Married or lives with partner	201596	119162 (59.1)	0.94 (0.93–0.95)	<0.01	0.87 (0.86–0.89)	<0.01
Education						
Middle school or above	231092	145738 (63.1)	1.00		1.00	
Primary school or below	145077	75502 (52.0)	1.57 (1.55–1.60)	<0.01	1.30 (1.28–1.32)	<0.01
Occupation						
Other*	210105	119033 (56.7)	1.00	<0.01	1.00	
Farmer or rural laborer	178391	102947 (57.7)	0.96 (0.95–0.97)		0.99 (0.97–1.00)	0.15
Ethnicity						
Minority group	117896	53500 (45.4)	1.00		1.00	
Han	270600	168480 (62.3)	0.50 (0.50–0.51)	<0.01	0.76 (0.74–0.77)	<0.01
Route of HIV infection						
Heterosexual contact	222148	143431 (64.6)	1.00		1.00	
Male-to-male sexual contact	44840	35277 (78.7)	0.49 (0.48–0.51)	<0.01	0.62 (0.60–0.64)	<0.01
Injection drug use	76815	26791 (34.9)	3.40 (3.34–3.46)	<0.01	2.07 (2.02–2.12)	<0.01
Sexual contact and injection drug use	5030	2111 (42.0)	2.52 (2.38–2.67)	<0.01	1.87 (1.76–1.99)	<0.01
Blood (plasma) donation	17204	10429 (60.6)	1.18 (1.15–1.22)	<0.01	0.83 (0.81–0.87)	<0.01
Site of HIV diagnosis						
VCT centers	110360	73316 (66.4)	1.00		1.00	
Hospitals	153367	87886 (57.3)	1.48 (1.45–1.50)	<0.01	1.91 (1.88–1.95)	<0.01
Detention centers	47218	14846 (31.4)	4.32 (4.22–4.42)	<0.01	1.75 (1.70–1.80)	<0.01
Others**	77551	45932 (59.2)	1.36 (1.34–1.39)	<0.01	1.42 (1.39–1.46)	<0.01
Migrant worker***						
No	294016	177081 (60.2)	1.00		1.00	
Yes	94480	44899 (47.5)	1.67 (1.65–1.70)	<0.01	1.55 (1.53–1.58)	<0.01
Total	388496	221980 (57.1)	-	-	-	-

*Includes laborer, unemployed, businessman, student, public servant, and unclear.

**Includes targeted intervention project, physical examination for sex workers, and unclear.

***Defined as having migrated from the registered region of residence to another region for at least six months.

In the univariate logistic regression model, factors associated with baseline CD4 cell count testing within 6 months of HIV diagnosis were age group, gender, marital status, education level, ethnicity, employment as a migrant worker, route of HIV transmission, site of HIV diagnosis, and year of HIV diagnosis (Table 2).

In the multivariate logistic regression model (Table 2), predictors for not receiving CD4 cell count testing with 6 months included being male (OR: 1.17, 95% CI: 1.15–1.19), age 55 years or older (OR: 1.03, 95% CI: 1.00–1.06), educational attainment of primary school or below (OR: 1.30, 95% CI: 1.28–1.32), occupation as a farmer or rural laborer (OR: 1.16, 95% CI: 1.15–1.18), route of HIV transmission classified as injecting drug use (OR: 2.07, 95% CI: 2.02–2.12) or sexual contact and injecting drug use (OR: 1.87, 95% CI: 1.76–1.99), HIV diagnosis in a hospital (OR: 1.91, 95% CI: 1.88–1.95) or a detention center (OR: 1.75, 95% CI: 1.70–1.80), and being a migrant worker (OR: 1.55, 95% CI: 1.53–1.58). Factors associated with timely CD4 testing included being married or cohabiting with a partner (OR: 0.87, 95% CI: 0.86–0.89), being of Han ethnicity (OR: 0.76, 95% CI: 0.74–0.77), and route of HIV transmission classified as male-to-male sexual contact (OR: 0.62, 95% CI: 0.60–0.64) or commercial blood plasma donation (OR: 0.83, 95% CI: 0.81–0.87).

Baseline CD4 cell counts were also analyzed by the route of HIV infection and the year of reporting (Table 3). There were significant differences in the distributions of CD4 cell counts by the routes of HIV infection and by the year of HIV diagnosis (heterosexual contact: χ^2^ = 119.63, p<0.01; male-to-male sexual contact: χ^2^ = 21.07, p<0.01; IDUs: χ^2^ = 191.85, p<0.01; and commercial blood plasma donation: χ^2^ = 66.95, p<0.01). Individuals infected through heterosexual contact and commercial blood plasma donation were more likely to have baseline CD4 cell counts <200 cells/µl than individuals infected by male-to-male sexual contact, injection drug use, or sexual contact and injection drug use.

**Table 3:** Number and percentage of newly HIV-diagnosed adults receiving baseline CD4 cell count testing within 6 months of diagnosis in China: 2006–2012, by routes of HIV transmission.

		2006		2007		2008		2009		2010		2011		2012		χ^2^
	Total	No.	%	No.	%	No.	%	No.	%	No.	%	No.	%	No.	%	P-value
Heterosexual contact																
<200	54579	1519	46.0	3043	42.0	4863	39.3	7229	39.7	9459	38.7	13277	37.7	15189	35.6	
200–349	35232	712	21.5	1686	23.2	3015	24.4	4279	23.5	6031	24.7	8870	24.7	10639	24.9	χ^2^ = 119.63
350–500	28918	522	15.8	1282	17.7	2298	18.6	3426	18.8	4674	19.1	7225	19.1	9491	22.3	p<0.01
≥500	24702	552	16.7	1240	17.1	2202	17.8	3274	18.0	4261	17.4	5839	17.4	7334	17.2	
Male-to-male sexual contact																
<200	6622	70	28.7	165	24.6	371	18.3	662	18.3	1059	18.8	1822	19.6	2473	18.0	
200–349	9274	65	26.6	182	27.1	575	28.4	1019	28.1	1525	27.0	2348	25.2	3560	25.9	χ^2^ = 21.07
350–500	10438	54	22.1	183	27.2	568	28.1	1033	28.5	1651	29.2	2763	29.7	4186	30.4	p<0.01
≥500	8943	55	22.5	142	21.1	511	25.2	910	25.1	1413	25.0	2383	25.6	3529	25.7	
Injection drug use																
<200	6635	549	33.1	867	30.5	1006	27.5	1115	26.4	1051	23.3	1100	21.4	947	19.9	
200–349	6158	375	22.6	660	23.2	840	23.0	991	23.5	1015	22.5	1209	23.5	1068	22.5	χ^2^ = 191.81
350–500	6277	305	18.3	601	21.1	802	22.0	901	21.3	1072	23.8	1312	25.5	1284	27.0	p<0.01
≥500	7721	431	26.0	715	25.2	1003	27.5	1213	28.8	1373	30.4	1530	29.7	1456	30.6	
Sexual contact and injection drug use																
<200	566	8	40.0	19	35.8	90	24.9	140	32.9	94	20.8	126	29.2	89	24.3	
200–349	482	5	25.0	10	18.9	95	26.2	86	20.2	98	21.7	92	21.3	96	26.2	χ^2^ = 0.85
350–500	461	3	15.0	7	13.2	78	21.5	86	20.2	106	23.5	89	20.6	92	25.1	p = 0.36
≥500	602	4	20.0	17	32.1	99	27.3	113	26.6	154	34.1	125	28.9	90	24.5	
Blood (plasma) donation																
<200	6502	1030	66.3	1215	68.3	1129	60.6	1046	63.2	824	61.4	773	56.5	485	55.8	
200–349	1867	274	17.6	290	16.3	364	19.5	281	17.0	241	17.9	247	18.1	170	19.6	χ^2^ = 66.95
350–500	1152	149	9.6	143	8.0	192	10.3	178	10.8	153	11.4	198	14.5	139	16.0	p<0.01
≥500	908	100	6.4	131	7.4	177	9.5	150	9.0	125	9.3	150	11.0	75	8.6	

The median baseline CD4 cell counts for all age groups increased slightly from 2006 to 2012 (Figure 1). However, the median baseline CD4 cell count for patients 45 years and older remained below 250 cells/µl over the study period. The median baseline CD4 cell counts of patients by route of transmission show none-to-little increase over the study period (Figure 2). Individuals infected through heterosexual contact and through commercial blood plasma donation had considerably lower median baseline CD4 cell counts than other subgroups.

**Figure 1:** Median baseline CD4 cell counts (within 6 months of diagnosis) of newly diagnosed HIV individuals in China from 2006 to 2012, stratified by age group. The median baseline CD4 cell counts, stratified by age group, increased each year from 2006 to 2012. Older age groups were associated with lower median baseline CD4 cell counts.

**Figure 2:** Median baseline CD4 cell counts (within 6 months of diagnosis) of newly diagnosed HIV individuals in China from 2006 to 2012, stratified by routes of infection. The median baseline CD4 cell counts, stratified by route of transmission, increased each year from 2006 to 2012. Subjects infected through injection drug use, male-to-male sexual contact, or sexual contact and injection drug use were consistently associated with higher median baseline CD4 cell counts compared to those infected through heterosexual contact or infected through blood (plasma) donation.

## Discussion

The aim of our study was to identify the proportion of HIV-positive individuals in China who received baseline CD4 testing within 6 months and characteristics associated with failing to receive testing within 6 months. CD4 cell count measurements are a standard component of HIV testing algorithms to monitor disease progression. Few past studies in China [20] have evaluated access to baseline CD4 cell count testing, and this is the first study to present results on a national scale.

In the era of “Treatment as Prevention,” early HIV detection, timely monitoring of disease progression, and early linkage to ART are critical steps to curbing the spread of HIV [25], [26], [27], [28]. In the United States, about 77% of HIV-diagnosed individuals are linked to care within 3–4 months, and 51% were retained in ongoing care [29]. With effective interventions such as the addition of case management, the proportion of HIV-positive patients linked to ongoing care can be significantly increased compared to those who receive the standard of care [30]. As China continues to develop and expand its national AIDS programs, including the NFATP, it will be critical to have regular assessment and monitoring of the programs' ability to link newly identified HIV-positive individuals to timely CD4 testing and treatment initiation.

To monitor the implementation of the national AIDS programs, NCAIDS developed annual quantitative targets of core program elements, including the “proportion of people known to be living with HIV whose CD4 cell counts were monitored at least once a year, to determine anti-retroviral therapy eligibility” [21]. For individuals nationwide diagnosed with HIV and AIDS, this proportion rose from 45.3 and 10.1% in 2007 to 54.2 and 62.5% in 2009, respectively [21]. Expanding on this previous finding, this current study shows that significant progress has also been made in increasing baseline CD4 cell count testing among HIV newly diagnosed individuals, as evidenced by the increase in CD4 cell count testing within 6 months from 20.0% in 2006 to 76.9% in 2012. The increases in CD4 monitoring of both new HIV cases and previously diagnosed cases were facilitated by structural expansions of the national AIDS programs and increases in the availability of testing materials/equipment [20], [31].

National policies recommend that the blood draw for the baseline CD4 cell count test should be completed at the first follow-up visit, which is scheduled at 14 days following the diagnosis. In our study, about 53.7% of individuals diagnosed in 2012 did not receive baseline CD4 cell count testing by the 14-day benchmark, and 23.1% did not receive CD4 cell count testing within 6 months. We identified several individual-level risk factors for failing to receive CD4 cell count testing within 6 months: age 55 years or older, male, primary school education or below, route of HIV transmission categorized as injection drug use or combined sexual contact and injection drug use, being diagnosed at a hospital or a detention center, and being a migrant worker. Some population-level factors are also likely to influence the obtainment and timing of CD4 testing. Until recent years, many county hospitals did not have the CD4 cell count testing equipment. In several regions with very low HIV prevalence, some counties and municipalities only had one CD4 detection machine for the entire area. This was likely to have delayed CD4 cell count testing for a small propotion of newly diagnosed HIV-positive individuals. Other population-level factors may include stigma and long distances between residences and clinics [32].

In our study, the majority of newly HIV diagnosed individuals were infected through heterosexual contact (Table 2). This is in accordance with recent literature indicating that sexual transmission has become the dominant mode of HIV transmission in China [23], [33], [34]. Over 60% of these individuals had baseline CD4 cell counts <350 cells/µl over the study period (Table 3), which is a higher proportion than those infected by male-to-male sexual contact or injection drug use. While HIV in China was historically driven by epidemics among injection drug users (IDUs), China will need to adjust to the challenges of facing an HIV epidemic that is predominantly spread by sexual contact. The group with the highest proportion (over 75%) of CD4 cell counts <350 cells/µl were individuals infected through commercial blood plasma donation. In the mid-1990s, there were major outbreaks of HIV through unsafe commercial blood and plasma donations [35], [36]. The extent of the epidemic was identified through large-scale targeted screening interventions among former paid plasma donors [37].

The two populations who had the highest median baseline CD4 counts were IDUs and men who have sex with men (MSM). This suggests that outreach efforts to reach these high-risk populations have produced some success in promoting early and regular HIV screening. However, MSM had the highest percentage of timely CD4 testing (78.7%) while IDUs had the lowest percentage (34.9%) when comparing subpopulations by route of transmission. Past research studies have similarly noted that MSM present with higher median CD4 levels compared to other risk groups [7]. In our study cohort, the relative success in linking HIV-positive MSM to timely CD4 testing may also be due to a comprehensive prevention and control program in sixty-one cities from 2008 to 2009 targeted towards MSM. This program was carried out with the support of MSM community groups. This program led to policies and additional ongoing intervention programs that address HIV prevention, HIV diagnosis and CD4 cell count testing among MSM.

The barriers for IDUs to access medical care are well-documented [38]. In China, many IDUs are engaged in migrant work, have unstable lifestyles, experience stigma and discrimination from health providers, and face the fear of arrest due to the illegality of drug use in China [19]. Our study noted a slight increase of CD4 cell count levels in IDUs over the study period. In recent years, several intervention measures been taken to decrease illicit drug use and to strengthen prevention and control of HIV transmission among IDUs [39], [40]. Another significant strategy for engaging the HIV-positive IDU population in regular care is to expand access to methadone maintenance treatment, which has been shown to independently promote linkage to HIV care and treatment [41].

Our study found that older patients were more likely to present at late disease stages, which has been noted previously in the literature [42]. There is currently very limited research [43], [44] on elderly HIV patients in China, who are not typically considered a vulnerable population for contracting HIV. According to data in CRIMS, the number of newly diagnosed individuals who were 55 years old or older has significantly increased in recent years [unpublished data, NCAIDS, 2013], as it has in the United States. Further studies are needed to explore issues related to the diagnosis and treatment of elderly HIV-positive patients in China.

Perhaps due to the implementation of the national AIDS programs [21] the proportion of patients with advanced HIV disease (CD4 count <200 cells/µl) has declined slightly since 2007. Of the 221,963 individuals who received timely baseline CD4 testing, the proportion of patients diagnosed late with HIV has declined slightly over the study period from 2006 to 2012. In our study cohort, 34.5% of individuals (N = 76580) had baseline CD4 counts of <200 cells/µl and 58.8% (N = 130434) had baseline CD4 counts of <350 cells/µl (Table 1). Late diagnosis and late ART initiation are strongly associated with negative health outcomes, including suboptimal CD4 increases with treatment, a high rate of opportunistic infections, and increased risk of mortality [45]. Early identification of HIV and prompt monitoring are critical to improving patient outcomes and reducing disease transmission.

Our study has several limitations. First, all data is reported by local providers and may have not been uploaded to the national databases in a timely manner. While providers and CDC staff review the data for completeness and accuracy, there may be some errors in the database. Second, in most cases, the route of infection was self-reported by the individual, and some misreporting may have occurred due to stigma, particularly for the categories of male-to-male sexual contact and injection drug use. Third, while we attempted to reduce the influence of confounding variables by using multivariate analysis, it remains possible that there was confounding by unmeasured variables. Fourth, our study analysis did not assess disease progression of the newly diagnosed HIV/AIDS patients by clinical staging or viral load testing. This information is available elsewhere in CRIMS; however, a full discussion of monitoring strategies over the study period is beyond the scope of this paper. Finally, our study did not exclude individuals who died between their diagnosis and the 6-month benchmark for timely CD4 testing. These patients were included in the 8% of the study cohort who were indicated as lost to follow-up and subsequently categorized as not having received timely CD4 testing. A study that only assesses individuals who were still living 6 months after HIV diagnosis may produce higher rates of timely CD4 testing.

The risk factors identified in this study should guide future intervention strategies to increase early HIV diagnosis and CD4 cell count testing among key populations. In recent years, an increasing number of HIV cases have been identified at VCT clinics at local CDC sites, which have higher rates of linkage to baseline CD4 testing. Regional strategies that have achieved success in reducing loss to follow up and increasing linkage to care have included in-parallel Western blot confirmation testing and baseline CD4 testing (Yunnan) and compressing the timeframe from screening, confirmation, and CD4 testing (Guangxi).

This study's evaluation of baseline CD4 cell count testing after HIV diagnosis provides a valuable reference for further increasing testing coverage and linkage to care. Despite significant improvement, a high proportion (23.1%) of HIV-positive patients still failed to receive timely CD4 count testing in 2012, the last year of the study. To shorten the time to CD4 cell count testing and to improve access to regular testing and treatment, there should be efforts to dramatically improve referrals and integration of patient tracking between the health facilities responsible for patient follow-up, CD4 cell count testing, and ART delivery.

## References

[1] MellorsJW, MuñozA, GiorgiJV, MargolickJB, TassoniCJ, et al (1997) Plasma viral load and CD4+ lymphocytes as prognostic markers of HlV-1 infection. Annals of Internal Medicine 126: 946–954.918247110.7326/0003-4819-126-12-199706150-00003

[2] HoggRS, YipB, ChanKJ, WoodE, CraibKJ, et al (2001) Rates of disease progression by baseline CD4 cell count and viral load after initiating triple-drug therapy. JAMA 286: 2568–2567.1172227110.1001/jama.286.20.2568

[3] DybulM, BolanR, CondoluciD, Cox-IyamuR, RedfieldR, et al (2002) Evaluation of initial CD4+ T cell counts in individuals with newly diagnosed human immunodeficiency virus infection, by sex and race, in urban settings. Journal of Infectious Diseases 185: 1818–1821.1208533210.1086/340650

[4] HammerSM, SquiresKE, HughesMD, GrimesJM, DemeterLM, et al (1997) A controlled trial of two nucleoside analogues plus indinavir in persons with human immunodeficiency virus infection and CD4 cell counts of 200 per cubic millimeter or less. AIDS Clinical Trials Group 320 Study Team. N Engl J Med 337: 725–733.928722710.1056/NEJM199709113371101

[5] ChaissonRE, KerulyJC, MooreRD (2000) Association of initial CD4 cell count and viral load with response to highly active antiretroviral therapy. JAMA 284: 3128–3129.1113577510.1001/jama.284.24.3128

[6] ChadbornTR, DelpechVC, SabinCA, SinkaK, EvansBG (2006) The late diagnosis and consequent short-term mortality of HIV-infected heterosexuals (England and Wales, 2000–2004). AIDS 20: 2371–2379.1711702410.1097/QAD.0b013e32801138f7

[7] BuchaczK, ArmonC, PalellaFJ, BakerRK, TedaldiE, et al (2012) CD4 Cell Counts at HIV Diagnosis among HIV Outpatient Study Participants, 2000–2009. AIDS Res Treat 2012: 869841.2194164010.1155/2012/869841PMC3176626

[8] OgbuanuIU, TorresME, KettingerL, AlbrechtH, DuffusWA (2009) Epidemiological characterization of individuals with newly reported HIV infection: South Carolina, 2004–2005. American Journal of Public Health 99 Suppl 1S111–117.1804878410.2105/AJPH.2006.104323PMC2724932

[9] GardnerEM, McLeesMP, SteinerJF, Del RioC, BurmanWJ (2011) The spectrum of engagement in HIV care and its relevance to test-and-treat strategies for prevention of HIV infection. Clinical Infectious Diseases 52: 793–800.2136773410.1093/cid/ciq243PMC3106261

[10] AlthoffKN, GangeSJ, KleinMB, BrooksJT, HoggRS, et al (2010) Late presentation for human immunodeficiency virus care in the United States and Canada. Clinical Infectious Diseases 50: 1512–1520.2041557310.1086/652650PMC2862849

[11] EasterbrookPJ, YuLM, GoetghebeurE, BoagF, McLeanK, et al (2000) Ten-year trends in CD4 cell counts at HIV and AIDS diagnosis in a London HIV clinic. AIDS 14: 561–571.1078071910.1097/00002030-200003310-00012

[12] CD4 Collaborative Group (1992) Use of monitored CD4 cell counts: predictions of the AIDS epidemic in Scotland. AIDS 6: 213–222.1348418

[13] ThanawuthN, ChongsuvivatwongV (2008) Late HIV diagnosis and delay in CD4 count measurement among HIV-infected patients in Southern Thailand. AIDS Care 20: 43–50.1827861410.1080/09540120701439303

[14] TranDA, ShakeshaftA, NgoAD, RuleJ, WilsonDP, et al (2012) Structural Barriers to Timely Initiation of Antiretroviral Treatment in Vietnam: Findings from Six Outpatient Clinics. PloS one 7: e51289.2324001310.1371/journal.pone.0051289PMC3519823

[15] KranzerK, ZeineckerJ, GinsbergP, OrrellC, KalaweNN, et al (2010) Linkage to HIV Care and Antiretroviral Therapy in Cape Town, South Africa. PloS one 5: e13801.2107219110.1371/journal.pone.0013801PMC2970551

[16] ZhangF, DouZ, MaY, ZhangY, ZhaoY, et al (2011) Effect of earlier initiation of antiretroviral treatment and increased treatment coverage on HIV-related mortality in China: a national observational cohort study. Lancet Infect Dis 11: 516–524.2160084910.1016/S1473-3099(11)70097-4

[17] Zhang F, Dou Z, Ma Y, Zhao Y, Liu Z, et al. (2009) Five-year outcomes of the China National Free Antiretroviral Treatment Program. Annals of Internal Medicine 151: : 241–251, W–252.10.7326/0003-4819-151-4-200908180-0000619687491

[18] WuZ, WangY, DetelsR, Rotheram-BorusMJ (2010) China AIDS policy implementation: reversing the HIV/AIDS epidemic by 2015. International Journal of Epidemiology 39 Suppl 2ii1–3.2111303110.1093/ije/dyq220PMC2992622

[19] ZhangF, HabererJE, WangY, ZhaoY, MaY, et al (2007) The Chinese free antiretroviral treatment program: challenges and responses. AIDS 21: S143–148.1817238310.1097/01.aids.0000304710.10036.2b

[20] ZhangY, LuL, LiHQ, LiuW, TangZR, et al (2011) Engaging HIV-infected patients in antiretroviral therapy services: CD4 cell count testing after HIV diagnosis from 2005 to 2009 in Yunnan and Guangxi, China. Chinese Medical Journal 124: 1488–1492.21740803

[21] LiuY, WuZ, MaoY, RouK, WangL, et al (2010) Quantitatively monitoring AIDS policy implementation in China. International Journal of Epidemiology 39 Suppl 2ii90–96.2111304210.1093/ije/dyq214PMC2992619

[22] WenY, ZhaoD, MaY, ZhaoY, LuL, et al (2011) Some patient-related factors associated with late access to ART in China' s free ART program. AIDS Care 23: 1226–1235.2193940210.1080/09540121.2011.555748

[23] DouZ, ChenRY, XuJ, MaY, JiaoJH, et al (2010) Changing baseline characteristics among patients in the China National Free Antiretroviral Treatment Program, 2002–09. International Journal of Epidemiology 39 Suppl 2ii56–64.2111303810.1093/ije/dyq215PMC2992620

[24] MaoY, WuZ, PoundstoneK, WangC, QinQ, et al (2010) Development of a unified web-based national HIV/AIDS information system in China. International Journal of Epidemiology 39 Suppl 279–89.10.1093/ije/dyq213PMC299261821113041

[25] GalvanFH, BingEG, BluthenthalRN (2000) Accessing HIV testing and care. Journal of Acquired Immune Deficiency Syndromes 25 Suppl 2S151–156.1125673610.1097/00042560-200012152-00010

[26] GarcíaF, de LazzariE, PlanaM, CastroP, MestreG, et al (2004) Long-term CD4+ T-cell response to highly active antiretroviral therapy according to baseline CD4+ T-cell count. Journal of Acquired Immune Deficiency Syndromes 36: 702–713.1516728910.1097/00126334-200406010-00007

[27] UNAIDS (2012) Global report 2012: UNAIDS report on the global AIDS epidemic. Geneva: UNAIDS.

[28] HullMW, WuZ, MontanerJS (2012) Optimizing the engagement of care cascade: a critical step to maximize the impact of HIV treatment as prevention. Curr Opin HIV AIDS 7: 579–586.2307612310.1097/COH.0b013e3283590617

[29] Centers for Disease Control and Prevention (CDC) (2011) Vital signs: HIV prevention through care and treatment—United States. MMWR Morbidity and Mortality Weekly Report 60: 1618–1623.22129997

[30] GardnerLI, MetschLR, Anderson-MahoneyP, LoughlinAM, del RioC, et al (2005) Efficacy of a brief case management intervention to link recently diagnosed HIV-infected persons to care. AIDS 19: 423–431.1575039610.1097/01.aids.0000161772.51900.eb

[31] JiangY, QiuM, ZhangG, XingW, XiaoY, et al (2010) Quality assurance in the HIV/AIDS laboratory network of China. International Journal of Epidemiology 39 Suppl 2ii72–78.2111304010.1093/ije/dyq224PMC2992624

[32] GovindasamyD, FordN, KranzerK (2012) Risk factors, barriers and facilitators for linkage to antiretroviral therapy care: a systematic review. AIDS 26: 2059–2067.2278122710.1097/QAD.0b013e3283578b9b

[33] WuZ (2011) New challenge and complex situation on HIV/AIDS control and prevention in China (in Chinese). Chin J Public Health 27: 1505–1507.

[34] WangN, WangL, WuZ, GuoW, SunX, et al (2010) Estimating the number of people living with HIV/AIDS in China: 2003–2009. International Journal of Epidemiology 39 Suppl 2ii21–ii28.2111303310.1093/ije/dyq209PMC2992614

[35] WuZ, LiuZ, DetelsR (1995) HIV-1 infection in commercial plasma donors in China. Lancet 346: 61–62.10.1016/s0140-6736(95)92698-47603178

[36] WuZ, SullivanSG, WangY, Rotheram-BorusMJ, DetelsR (2007) Evolution of China's response to HIV/AIDS. Lancet 369: 679–690.1732131310.1016/S0140-6736(07)60315-8PMC7137740

[37] WuZ, RouK, DetelsR (2001) Prevalence of HIV infection among former commercial plasma donors in rural eastern China. Health Policy and Planning 16: 41–46.1123842910.1093/heapol/16.1.41

[38] CelentanoDD, GalaiN, SethiAK, ShahNG, StrathdeeSA, et al (2001) Time to initiating highly active antiretroviral therapy among HIV-infected injection drug users. AIDS 15: 1707–1715.1154694710.1097/00002030-200109070-00015

[39] YinW, HaoY, SunX, GongX, LiF, et al (2010) Scaling up the national methadone maintenance treatment program in China: achievements and challenges. International Journal of Epidemiology 39 Suppl 2ii29–37.2111303410.1093/ije/dyq210PMC2992615

[40] SmithK, BartlettN, WangN (2012) A harm reduction paradox: comparing China's policies on needle and syringe exchange and methadone maintenance. Int J Drug Policy 23: 327–332.2237734110.1016/j.drugpo.2011.09.010PMC7135432

[41] Zhao Y, Shi CX, McGoogan JM, Rou K, Zhang F, et al.. (2013) Predictors of accessing antiretroviral therapy among HIV-infected drug users in China's National Methadone Maintenance Treatment Program. Addiction Forthcoming.10.1111/add.12782PMC559617425533863

[42] MugaveroMJ, CastellanoC, EdelmanD, HicksC (2007) Late diagnosis of HIV infection: the role of age and sex. American Journal of Medicine 120: 370–373.1739823510.1016/j.amjmed.2006.05.050PMC3184035

[43] LiuH, LinX, XuY, ChenS, ShiJ, et al (2012) Emerging HIV epidemic among older adults in Nanning, China. Aids Patient Care and STDS 26: 565–567.2298477910.1089/apc.2012.0227PMC3462385

[44] ChenX, ZhengJ, HeJM, QinB, HuY, et al (2011) Unusual increase in reported HIV/AIDS cases among older persons in western Hunan province, China. Sexually Transmitted Infections 87: 538.2187347110.1136/sextrans-2011-050228

[45] LawnSD, LittleF, BekkerLG, KaplanR, CampbelE, et al (2009) Changing mortality risk associated with CD4 cell response to antiretroviral therapy in South Africa. AIDS 23: 335–342.1911487010.1097/QAD.0b013e328321823fPMC3776050

